The article "Gu-Ben-Zhi-Ke-Zhong-Yao Alleviated PM2.5-Induced Lung Injury via HMGB1/NF-κB Axis" was retracted in 2023. Reasons: signs of a paper mill; suspected computer-generated content; unreliable results or conclusions; concerns about the data.

# Gu-Ben-Zhi-Ke-Zhong-Yao Alleviated PM2.5-Induced Lung Injury via HMGB1/NF-*κ*B Axis

**DOI:** 10.1155/2022/8450673

**Published:** 2022-03-30

**Authors:** Wenxiao Hou, Hongchun Zhang, Meng Jiang, Yina Wu, Tao Li, Luhong Cong, Jun Duan

**Affiliations:** ^1^Graduate School of Beijing University of Traditional Chinese Medicine, Beijing 100029, China; ^2^Surgical Intensive Care Unit, China Japan Friendship Hospital, Beijing 100029, China; ^3^Department of Health Care, China Japan Friendship Hospital, Beijing 100029, China; ^4^National Respiratory Center, Beijing 100029, China; ^5^Yunnan University of Traditional Chinese Medicine, Kunming 650011, China; ^6^Department of Emergency, China Japan Friendship Hospital, Beijing 100029, China

## Abstract

**Background:**

Inhalation of particles with a diameter of less than 2.5 *μ*m (PM2.5) among air pollutants may cause lung damage. Gu-Ben-Zhi-Ke-Zhong-Yao (GBZK) is a traditional Chinese medicine prescription that has a beneficial effect on the treatment of chronic obstructive pulmonary disease (COPD). However, the effect of GBZK on PM2.5-induced lung injury remains to be elucidated.

**Methods:**

We constructed a mice lung injury model through PM2.5 stimulation and simultaneously performed GBZK gavage treatment. After 4 weeks, the lung tissues of the mice were collected for pathological staining to analyze the degree of damage. The activities of myeloperoxidase (MPO), malondialdehyde (MDA), and oxidative stress-related factors (superoxide dismutase, SOD; glutathione peroxidase, GSH-Px) were detected by commercial kit in lung tissue. Furthermore, the number of neutrophils and related inflammatory factors (interleukin-1, IL-1*β*; tumor necrosis factor *α*, TNF-*α*; interleukin-6, IL-6) in bronchoalveolar lavage fluid (BALF) and serum were collected and tested to evaluate the effect of GBZK on inflammation. Masson staining was used to detect the level of lung fibrosis in mice. The activation of HMGB1 (high-mobility group protein 1) and NF*κ*Bp65 (nucleus factor kappa B) in lung tissue was evaluated by immunohistochemistry and western blot.

**Results:**

The result revealed that PM2.5 induces lung damage, and GBZK gavage treatment could reduce the degree of injury in a concentration-dependent manner in mice. After GBZK treatment, the MPO activity, MDA content, and oxidative stress level in the lung tissues of mice decreased. And after GBZK treatment, the expression levels of inflammatory cytokines in BALF and blood were decreased. GBZK treatment also improved pulmonary fibrosis in mice. In addition, we also found that GBZK prevented the up-regulation of the HMGB1/NF-*κ*B axis in the lungs of mice.

**Conclusion:**

These results indicated that GBZK might protect mice from PM2.5-induced lung injury by inhibiting the HMGB1/NF*κ*B pathway, thus repressing inflammation and pulmonary fibrosis.

## 1. Introduction

Air pollution is mainly due to excessive emissions of industrial waste gas and automobile exhaust and has become one of the main causes of respiratory diseases [1]. Among them, suspended particulate matter (PM) in the atmosphere is considered the most representative air pollutant, especially inhalable particulate matter (diameter ≤10 *μ*m) and fine particles (diameter ≤2.5 *μ*m, PM2.5) [2]. Long-term exposure to inhalable particles in the environment may pose a serious threat to human health [3]. Especially for PM2.5, it can enter the alveoli through the human respiratory tract, part of which remains in the lungs and causes respiratory tract infection, and the other part circulates into the human body through the bloodstream, leading to cardiovascular disease, systemic inflammation, and even lung cancer [4]. When a large amount of PM2.5 accumulates in the lungs, lung epithelial cells are repeatedly damaged, leading to pulmonary fibrosis [5]. At the same time, alveolar macrophages release excessive inflammatory factors to cause lung injury [6].

Gu-Ben-Zhi-Ke-Zhong-Yao (GBZK) is a Chinese herbal formula developed by Prof. Chao Enxiang according to the pathological characteristics of chronic obstructive pulmonary disease (COPD), based on three traditional Chinese medicines: Astragalus, Fangfeng, and Atractylodes [7]. The use of GBZK in the clinical treatment of COPD patients shows extremely effective, and there are no obvious side effects [8]. Furthermore, animal experiments have also shown that GBZK has a good effect on maintaining the integrity of the airway wall and promoting the repair of lung inflammation [9]. However, the regulatory mechanism of GBZK in lung injury, especially PM2.5-induced lung injury, is still unclear.

High-mobility group box-1 protein (HMGB1) is a highly conserved nuclear DNA binding protein that can participate in the inflammatory response [10]. As a late-stage inflammatory cytokine, the up-regulation of HMGB1 can cause an excessive inflammatory response by stimulating cells to produce inflammatory factors [11]. Inhibiting the expression of HMGB1 in acute lung injury was proved to reduce inflammation and tissue damage [12, 13]. Inhibiting the expression of HMGB1 in acute lung injury (Ali) was proved to reduce inflammation and tissue damage via regulating NF-*κ*B signaling [14, 15]. The study of Yu-Xiang Fei et al found that Ma Xing Shi Gan decoction inhibits HMGB1 in vivo and in vitro to reduce PM2.5-induced inflammation and acute lung injury [3]. However, it has not been reported whether GBZK can improve PM2.5-induced acute lung injury by inhibiting HMGB1.

This research aims to confirm the therapeutic effect of GBZK on lung damage caused by PM-2.5 and its possible molecular mechanism and develop a new and safe treatment plan for lung injury caused by PM-2.5.

## 2. Materials and Methods

### 2.1. Preparation of GBZK

The traditional Chinese medicine for consolidating cough was composed of Astragalus, Fructus Anemarrhena, Atractylodes macrocephala, Epimedium, Bupleurum, Scutellaria baicalensis Georgi, and Radix Paeoniae and purchased from China-Japan Friendship Hospital. The medicine was made into a dry extract by the preparation room of China-Japan Friendship Hospital, Beijing, China, which contained 4g of crude drug per milliliter. In the experiment, it was configured to three concentrations of 0.2, 0.4, 0.8 g crude drug/ml.

### 2.2. Purchase and Breeding of Animals and Establishment of PM2.5-Induced Lung Injury Model

50 adult female BLAB/c mice (18–25g) were purchased from Beijing MaiDeKangNa Biotechnology Company. Food and water were provided for breeding in the SPF level laboratory in accordance with the breeding standards. According to the experimental requirements, the mice were divided into 5 groups: control, PM2.5, PM2.5+GBZK L (8 g/kg/day), PM2.5+GBZK M (16 g/kg/day), and PM2.5+GBZK H (32 g/kg/day).

PM2.5 samples were collected from March 2021 to April 2021 using an air sampler on the open roof of a 10-story building at the China-Japan Friendship Hospital, Beijing. To decontaminate, the filters were preheated to 550°C. Then, they were equilibrated and stabilized (20 ± 0.5°C, 40 ± 5% RH) before sampling. The filters containing the samples were cut into 1 cm × 1 cm sizes, immersed in sterilized ddH2O, and eluted by ultrasonic shock three times. The eluate was filtered through medical gauze and then freeze-dried in a vacuum freeze-dryer and sealed at −80°C for storage. Before use, PM2.5 particles were prepared in phosphate-buffered saline (PBS) to a concentration of 10 mg/mL particle suspension.

Except for the control group, mice in the other four groups were exposed to PM2.5 stimulation for 4 weeks via a continuous intranasal drip of PM2.5 (7.5 mg/kg body weight/day) and were given different concentrations of GBZK gavage for 4 weeks at the same time. The control group was given the same amount of normal saline.

All animal-related experiments had been approved by the ethics committee of China-Japan Friendship Hospital, Beijing, China.

### 2.3. Hematoxylin-Eosin (HE) Staining Analysis

Briefly, lung tissue with a thickness of no more than 0.5 cm was put into a preprepared fixative (10% formalin, Bouin's fixative, etc.) for tissue fixation. Then, we used different concentrations of alcohol, xylene, and paraffin to dehydrate and embed the tissue blocks and made paraffin sections. Then, xylene was used for dewaxing, and the section was rinsed with alcohol and distilled water 5 times and then dyed with hematoxylin for 5 min. Next, the slices were flushed with deionized water and dyed with eosin for 1 min. The slices were dehydrated with ethanol, and then, xylene was added. Finally, the slides were fixed, and the section was analyzed under a microscope.

### 2.4. Lung Wet to Dry Ratio (W/D)

The mouse lung tissue was collected and weighed, the tissue was dried in an oven at 80 °C for 36 h, and the dry weight was weighed.

### 2.5. Analysis of MPO Activity and MDA Content

0.1 g lung tissue from mice was collected, and the MPO level was detected employing the myeloperoxidase (MPO) fluorometric activity assay kit (BioVision, K745-100, USA) according to the instructions. The MDA content in the tissues was detected using a malondialdehyde (MDA) content detection kit (Solarbio, BC0020, China).

### 2.6. Analysis of SOD and GSH-Px Activity

Mice lung tissue samples were tested for SOD activity using the total SOD activity detection kit (WST-8 method) (Beyotime, S0101S, China) according to the instructions. The mice glutathione peroxidase (GSH-Px) ELISA test kit (Laibio, JL20363, China) was used to detect the GSH-Px activity in the sample.

### 2.7. BALF to Detect the Total Cell Level of BALF and the Level of Neutrophils

3 ml blood from mice's abdominal aorta was subjected to 2800 g and centrifuged for 20 min, and the serum was collected. Through the mice trachea was intubated, the left lung was washed 3 times with 0.5 mL of iced PBS, and then, BALF was collected. The collected sample was centrifuged at 800 g for 10 min. The cell pellet obtained by centrifugation was suspended in 100 *µ*L PBS, and the total cell number was measured with a hemocytometer (Shanghai Qiujing, China). The cell was dyed with Wright-Giemsa (Rongbio, RBR00502, China) for 10 min. Finally, the different cells were counted through an optical microscope.

### 2.8. ELISA to Detect Inflammatory Factors

In accordance with the requirements of the instructions, the levels of inflammatory factors were detected by ELISA kits. In accordance with requirements of the instructions, the levels of inflammatory factors (IL-1*β*, TNF-*α*, and IL-6) were detected by Mouse (IL-1*β*) ELISA Kit (sbjbio, SBJ_M0583, China), Mouse Tumor Necrosis Factor *α* (TNF-*α*) ELISA Kit (sbjbio, SBJ-M0030-96T, China), and Mouse Interleukin 6 (IL-6) ELISA kit (sbjbio, SBJ-M0044, China).

### 2.9. Masson Stain

The paraffin sections of mice lung tissues were deparaffinized. After rinsing the slices with deionized water, the slices were dyed with Regaud's hematoxylin dye solution and rinsed with distilled water 5 times after 10 min. The sections were then treated with Masson's ponceau acid fuchsin for 8 min. Afterwards, it was soaked in the 2% glacial acetic acid aqueous (GAA) solution for 5 min, and a 1% phosphomolybdic acid aqueous solution was added to differentiate the slices. After 5 min, the sections were directly stained with aniline blue for 5 min. Finally, the slices were soaked in the 0.2% GAA aqueous solution for 5 min, then sealed with anhydrous alcohol, xylene, and neutral gum, and observed under an optical microscope.

### 2.10. Immunohistochemistry

First, the paraffin sections of mice lung tissues were deparaffinized. The sections were incubated for 8 min in 3% H_2_O_2_ at room temperature, then rinsed with distilled water 3 times, and soaked in PBS for 5 min. Then, 10% normal goat serum was used to block the sections for 10 min at room temperature. Section and primary antibody *α*-SMA (ab232784, Abcam, UK) and collagen I (ab270993, Abcam, UK) were incubated overnight at 4 °C and washed with PBS 3 times. Then, the biotin-labeled secondary antibody was added to the slices and incubated at 37 °C for 30 min. Then, it was rinsed 3 times with PBS, and the sections were incubated with horseradish enzyme-labeled streptavidin for 30 min at room temperature. Finally, diaminobenzidine was used to color the sections, and the sections were counterstained with hematoxylin. The staining results were observed and recorded through an optical microscope.

### 2.11. Western Blot

First, the mice lung tissues were lysed with RIPA lysis buffer. Bicinchoninic acid (BCA) was used to detect total protein. Then, the same amount of protein was separated by 10% SDS-PAGE, and the protein band was transferred to the polyvinylidene fluoride (PVDF) membrane. After washing with TBST buffer, it was blocked with 5% skimmed milk for 2 h, incubated with primary antibody *α*-SMA (ab232784, Abcam, UK), collagen I (ab270993, Abcam, UK), HMGB1 (ab18256, Abcam, UK), p-NF-*κ*Bp65 (ab 183559, Abcam, UK), *ß*-actin (ab8226, Abcam, UK) at 4°C overnight, and washed 3 times with PBS. Then, it was incubated with HRP-conjugated anti-rabbit IgG secondary antibody for 2 h at room temperature. Finally, an enhanced chemiluminescence (ECL) solution (Millipore, USA) was added for development. ImageJ 1.50 was used for quantitative analysis.

### 2.12. Statistical Analysis

All data shown were average ± SD from three independent experiments, and GraphPad Prism 5.0 (GraphPad Software, La Jolla, CA, USA) software was used for data analysis. The one-way analysis of variance (ANOVA) was used for difference analysis, and Tukey's post hoc test was used for comparison between multiple groups. *p* < 0.05 was statistically significant.

## 3. Results

### 3.1. GBZK Attenuates PM2.5-Induced Lung Injury

First, in order to verify the effect of GBZK on lung injury, we constructed a lung damage mice model caused by PM-2.5. Three different concentrations (0.2, 0.4, and 0.8 ml/d) of GBZK were administered to the injured mice by gavage. After 4 weeks, the mice lung tissues were collected for HE staining (Figure 1(a)). All the lung structures in the PM-2.5 treatment group including bronchioles, alveoli, and pulmonary blood vessels were severely injured, mainly manifested as thickening of alveolar adventitia, hemorrhage, and pulmonary edema, compared with the control. With the increase of the treatment concentration of GBZK, the pathological change of lung tissue gradually reduced. Moreover, in the GBZK treatment group, the lung injury score was obviously lower than the PM-2.5 stimulation group (Figure 1(b)). Further test of the lung wet-to-dry ratio found that the lung water content increased visibly after PM-2.5 treatment, while the lung wet-to-dry ratio of GBZK treatment decreased, especially a concentration of 0.8 ml/d treatment was the most significant (Figure 1(c)). The above results suggested that GBZK alleviated PM-2.5-induced lung damage.

### 3.2. GBZK Attenuates PM2.5-Induced Oxidative Stress

We further analyzed the oxidative stress-correlative proteins (MPO, MDA, SOD, and GSH-Px) in mice lung tissue to evaluate the effect of GBZK on the degree of oxidative stress in lung tissue. PM-2.5 induced an increase in MPO and MDA activity in lung tissues, and after GBZK treatment, MPO and MDA activity reduced in a concentration-dependent manner (Figures 2(a) and 2(b)). Finally, the levels of SOD and GSH-Px were detected, and it was shown that the levels of SOD and GSH-Px in the PM-2.5-induced group were reduced, and the levels of SOD and GSH-Px were raised after the GBZK treatment (Figures 2(c)–2(d)). The above results show that GBZK attenuated the oxidative stress of lung tissue caused by PM-2.5.

### 3.3. GBZK Attenuates PM2.5-Induced Inflammatory Response

In order to explore the regulation of GBZK on the inflammatory response of mice lung tissue, we first collected mice blood and BALF and counted the total cell level and neutrophil level. The quantity of total cells and neutrophils in the BALF induced by PM-2.5 increased, while GBZK treatment substantially reduced the quantity of total cells and neutrophils (Figures 3(a) and 3(b)). Detecting the levels of inflammatory factors (IL-1*β*, TNF-*α*, IL-6) in the blood of mice by ELISA showed that PM-2.5 induced the expressions of inflammatory factors in the blood, while the expression levels of inflammatory factors were reduced after the GBZK treatment (Figures 3(c)–3(e)). Further detection of the expression levels of inflammatory factors in BALF found that, consistent with the levels in blood, PM-2.5 induced the expression levels of inflammatory factors in BALF, while GBZK treatment decreased the blood of inflammatory factors (Figures 3(f)–3(h)). In summary, the result revealed that GBZK attenuated PM-2.5-induced inflammatory response in mouse.

### 3.4. GBZK Attenuates PM2.5-Induced Pulmonary Fibrosis

We further analyzed the impact of GBZK on PM-2.5-induced lung fibrosis in mice. First, we used Masson staining to detect the level of mice lung fibrosis. PM-2.5 induced fibrosis in the mice lung tissue, with a large amount of collagen fiber deposition and lung interstitial thickening (Figure 4(a)). After GBZK treatment, the PM-2.5-induced fibrosis process was inhibited, and the accumulation of collagen fibers in the lung tissue was reduced (Figure 4(a)). Fiber marker (*α*-further immunohistochemical and Western blot analysis of SMA and type I collagen) showed that PM-2.5 could induce the upregulation of fibronectin expression in mouse lung tissue. However, the expressions of fibrosis marker proteins in lung tissues were suppressed after GBZK treatment (Figures 4(b) and 4(c)). In summary, we found that GBZK ameliorated PM-2.5-induced lung fibrosis.

### 3.5. GBZK Inhibits PM2.5-Induced HMGB1/NF-Κb Pathway

Finally, we tested the expression level of HMGB1 and the activation of NF-*κ*B to verify whether GBZK could improve PM-2.5-induced lung damage by regulating the HMGB1/NF-*κ*B axis. Immunohistochemical detection displayed that PM-2.5 induced the level of HMGB1 and phosphorylation of NF-*κ*Bp65 subunit in mice lung tissues. GBZK treatment significantly reduced PM-2.5-induced HMGB1 expression and NF-*κ*Bp65 phosphorylation (Figure 5(a)). Western blot further validated that PM-2.5 induced the level of HMGB1 and phosphorylation of NF-*κ*Bp65, and GBZK treatment reversed this effect (Figure 5(b)). In short, our tests revealed that GBZK inhibited PM-2.5-induced HMGB1/NF-*κ*B axis in mice lung tissue.

## 4. Discussion

According to statistics from the World Health Organization, 3.8 million people died of air pollution in 2015 [16]. PM2.5 enters the lungs with humans inhaling contaminated air. Some particles in PM2.5 may cause a variety of cracking reactions to produce free radicals, and these free radicals lead to cell peroxidation and inflammation [17]; on the other hand, alveolar macrophages release inflammatory factors by engulfing PM2.5 [18, 19]. These reasons directly cause the occurrence of inflammatory reaction, which leads to lung injury [20, 21]. Our verification confirmed in mice experiments that PM-2.5 caused lung injury in mice and induced oxidative stress, inflammation, and pulmonary fibrosis in lung tissue.

GBZK has been confirmed in clinical and animal studies to improve lung injury [7]. Previous studies have confirmed that the three main components of GBZK, Astragalus, Fangfeng, and Atractylodes can show protective and therapeutic effects in acute lung injury rats [22–24]. In particular, it has the most significant effect on reducing oxidative stress and inflammatory factors in rats with lung injury. Our study in mice also further confirmed the alleviative effect of GBZK on PM-2.5-induced lung damage. Our research not only confirmed that GBZK improved the release of oxidative stress and inflammatory factors in the lung tissue of mice induced by PM-2.5 but also found that GBZK could improve PM-2.5-induced pulmonary fibrosis in mice.

HMGB1 is a pro-inflammatory factor that may be released by macrophages or necrotic cells [25–27]. HMGB1 in the cytoplasm can cause lung injury and cancer by activating its downstream inflammatory pathways [28–31]. It has been claimed that the HMGB1 and NF*κ*B signaling pathways are activated in the lung damage tissue induced by PM2.5 stimulation in rats [3]. The NF-*κ*B signaling was proved to promote the expression of pro-inflammatory genes in the inflammatory response and is a key pathway for immune regulation [32]. HMGB1 can activate the NF-*κ*B pathway directly or indirectly to promote the release of inflammatory factors [33–35]. In our study, we consistently found that PM-2.5 induction could promote HMGB1 and release and activation of NF-*κ*B. After GBZK treatment, the content of HMGB1 in mice lung tissues decreased, and the activation of NF-*κ*B was inhibited. We speculated that GBZK might treat lung damage via the HMGB1/NF-*κ*B axis.

Chinese herb formula focuses on the patient and enhances the body's natural activity in a dialectical manner. In contrast, Western medicine focuses on the symptoms of the disease. The strength of the Chinese herb formula lies in the individualized and comprehensive consideration of treatment. However, the Chinese herb formula is often complex and contains multiple components. A weakness of the Chinese herb formula may be the difficulty of target identification; furthermore, even if efforts are being made to uncover the pharmacological mechanisms of Chinese herb formula, the mechanisms involved may not be easily and fully elucidated. Studies have shown lung injury protective effects of Chinese herb formula, including acute lung injury and COVID-19 [36, 37]. However, most of them have focused on inflammatory cytokines, oxidative stress, and inflammatory cell infiltration. Moreover, the material basis of the pharmacological effects of antilung injury should be clarified to provide a scientific basis for the prevention and treatment of lung injury by Chinese herb formula.

In conclusion, this study showed that GBZK prevented PM-2.5-induced lung damage by suppressing oxidative stress, the release of inflammatory factors, and the production of lung fibrosis. And the alleviative mechanism of GBZK might be connected with the suppression of the HMGB1/NF-*κ*B axis. Our research provided a new strategy for the prevention and treatment of lung injury.

## Figures and Tables

**Figure 1:** GBZK attenuates PM2.5-induced lung injury. A PM2.5-induced lung injury model in mice was constructed, and GBZK was administered for treatment. (a) Assessment of lung tissue damage by HE staining. (b) Lung histologic injury score. (c) The effect of GBZK on the lung wet-to-dry ratio induced by PM2.5. n = 10, ^*∗*^*p* < 0.05, ^*∗∗*^*p* < 0.01, ^*∗∗∗*^*p* < 0.001.

**Figure 2:** GBZK attenuates PM2.5-induced oxidative stress. (a) The effect of GBZK on MPO activity in lung tissue. (b) The effect of GBZK on MDA content in lung tissue. (c) The kit detected the activity of SOD and (d) GSH-Px in lung tissue. n = 10, ^*∗*^*p* < 0.05, ^*∗∗*^*p* < 0.01, ^*∗∗∗*^*p* < 0.001.

**Figure 3:** GBZK attenuates PM2.5-induced inflammatory response. Mice serum and BALF are collected. (a)-(b) The effect of GBZK on the total cell level and neutrophil level in BALF. (c)-(d)-(e) ELISA detected serum levels of IL-1*β*, TNF-*α*, and IL-6. (f)-(g)-(h) ELISA detected the levels of IL-1*β*, TNF-*α*, and IL-6 in BALF. *n* = 10, ^*∗*^*p* < 0.05, ^*∗∗*^*p* < 0.01, ^*∗∗∗*^*p* < 0.001.

**Figure 4:** GBZK attenuates PM2.5-induced pulmonary fibrosis. (a) Masson staining to detect the level of lung fibrosis in mice. (b) Immunohistochemical staining to detect the expression of *α*-SMA and collagen I in lung tissue. (c) Western blotting detects the expression of *α*-SMA and collagen I in lung tissue. n = 10, ^*∗*^*p* < 0.05, ^*∗∗*^*p* < 0.01, ^*∗∗∗*^*p* < 0.001.

**Figure 5:** GBZK inhibits PM2.5-induced HMGB1/NF-*κ*B pathway. (a) Immunohistochemical staining was used to detect the expression of HMGB1 and the phosphorylation level of NF-*κ*Bp65 in lung tissue. (b) Western blot detection of HMGB1 expression and NF-*κ*Bp65 phosphorylation level in lung tissue. n = 10, ^*∗*^*p* < 0.05, ^*∗∗*^*p* < 0.01, ^*∗∗∗*^*p* < 0.001.

## Data Availability

The data used to support the findings of this study are available from the corresponding author upon request.

## Abbreviations

PM2.5: Particles with a diameter of less than 2.5 *μ*m
COPD: Chronic obstructive pulmonary disease
GBZK: Gu-Ben-Zhi-Ke-Zhong-Yao
MPO: Myeloperoxidase
MDA: Malondialdehyde
BALF: Bronchoalveolar lavage fluid
HMGB1: High-mobility group box-1 protein
NIH: National Institutes of Health
BCA: Bicinchoninic acid
PVDF: Polyvinylidene fluoride
ECL: Chemiluminescence.
